# LncRNA OIP5-AS1 inhibits the lipopolysaccharide-induced inflammatory response and promotes osteogenic differentiation of human periodontal ligament cells by sponging miR-92a-3p

**DOI:** 10.1080/21655979.2022.2067291

**Published:** 2022-05-12

**Authors:** Shiwei Wang, Yao Duan

**Affiliations:** a Dental Department, The First Affiliated Hospital of Xi’an Medical University, Xi’an, Shanxi 710077, P.R. China; b Second Clinical Division, Peking University School and Hospital of Stomatology & National Clinical Research Center for Oral Diseases, National Engineering Laboratory for Digital and Material Technology of Stomatology & Beijing Key Laboratory of Digital Stomatology, Beijing 100081, P.R. China

**Keywords:** Long non-coding RNA OIP5 antisense RNA 1, human periodontal ligament cells, microRNA-92a-3p, periodontitis, osteogenic differentiation, inflammation

## Abstract

Periodontitis is a chronic infectious disease that affects the oral health of adults. Long non-coding RNA OIP5 antisense RNA 1 (OIP5-AS1) has been reported to downregulated in the periodontal tissue of patients with periodontitis. Therefore, the study sought to look at the possible functions of OIP5-AS1 in periodontitis and the associated underlying mechanisms. In the present study, the expression level of OIP5-AS1 and microRNA-92a-3p were analyzed using reverse transcription-quantitative PCR. The levels of osteogenic proteins were determined using western blotting and inflammatory cytokines and oxidative stress were also examined. The proliferation of human periodontal ligament stem cells (hPDLSCs) was evaluated using MTT assays. Assay of osteogenic differentiation was undertaken by means of Alkaline phosphatase staining. The possible association between OIP5-AS1 and miR-92a-3p was determined applying dual-luciferase reporter assays and verified by RNA immunoprecipitation assay. We found that OIP5-AS1 was expressed at low levels in lipopolysaccharide (LPS)-stimulated hPDLSCs. OIP5-AS1 overexpression promoted proliferation and osteogenic differentiation ability and reduced LPS-induced inflammation in hPDLSCs. Furthermore, OIP5-AS1 directly targeted and reduced miR-92a-3p expression. The overexpression of miR-92a-3p partly abolished the effects of OIP5-AS1 on LPS-induced cell proliferation and osteogenic differentiation as well as inflammation in hPDLSCs. Collectively, the results indicated that OIP5-AS1 overexpression inhibited the LPS-induced inflammatory response and promoted the osteogenic differentiation of hPDLSCs by sponging miR-92a-3p. Thus, OIP5-AS1 is probably an essential objective for research during periodontitis treatment.

## Highlights

- OIP5-AS1 overexpression promotes the proliferation and osteogenic differentiation, represses inflammation of hPDLSCs following LPS treatment.
- OIP5-AS1 directly targets miR-92a-3p.
- miR-92a-3p overexpression reverses the effect of OIP5-AS1 on the proliferation, osteogenic differentiation and inflammation of LPS-stimulated hPDLSCs.

## Introduction

Periodontitis is a chronic infectious disease involving multiple contributing factors, such as dental plaque and calculus [1,2]. Periodontitis is characterized by tooth mobility and bleeding from the gingival tissue that leads to the progressive destruction of the periodontium. Periodontitis leads to tooth loss and affects chewing function of adults [3]. Previous studies have demonstrated that the risk of developing periodontitis is affected by systemic diseases, like diabetes mellitus and osteoporosis, and environmental factors, like smoking and psychological stress [4–7]. Periodontal diseases impact ~90% of the global population [8]. Periodontitis and associated tooth loss cause considerable inconvenience to the patient and pose a threat to their overall health, thus, the development of an effective approach to treat periodontitis is required.

The osteogenic potential of human periodontal ligament stem cells (hPDLSCs) is commonly used for the self-renewal of periodontal tissue and the repair an degeneration of periodontally diseased tissues [9]. Thus, hPDLSCs have the ability to repair periodontal defects. Previous studies have reported that the inflammatory microenvironment decreases the osteogenic differentiation capacity of hPDLSCs [10,11]. Therefore, improving the osteogenic ability of hPDLSCs may act as promising therapeutic strategy for the treatment of periodontitis.

In previous years, research has concentrated on two types of non-coding RNAs, microRNAs (miRNAs/miRs) and long non-coding (lnc)RNAs, which play key regulatory roles in the pathogenesis of a number of inflammatory diseases [12–15]. LncRNAs play crucial roles in the occurrence and development of periodontitis and they can function as ceRNA to bind with miRNA to regulate downstream genes [16,17]. The results of a previous study demonstrated that the expression level of lncRNA OIP5-AS1 was downregulated in the periodontal samples of patients with gingivitis and periodontitis, compared with healthy subjects [18]. These findings suggested that OIP5-AS1 may act as an anti-inflammatory factor in systemic inflammation. However, there has been no detailed investigation of effect of OIP5-AS1 in periodontitis.

In the present study, we aimed to identify the role and mechanism of OIP5-AS1 in the inflammatory response of hPDLSCs and highlighted the importance of OIP5-AS1 in the therapy of periodontitis. LPS is a well-established potent stimulator of inflammation that promotes the secretion of inflammatory cytokines TNF-α, IL-6 and IL-1β [19–21]. In the present study, an in vitro model of periodontitis was established using hPDLSCs stimulated with different concentrations of LPS. We made the conjecture that OIP5-AS1 overexpression plays a beneficial role in LPS-stimulated hPDLSCs by targeting miR-92a-3p.

## Materials and methods

### Cell culture and transfection

Human periodontal ligament stem cells (hPDLSCs) were purchased from the American Type Culture Collection and cultured as previously described [22]. The third generation to the fifth generation of hPDLSCs was used in the present study and were maintained in minimum essential medium α (α-MEM; Gibco, Waltham, MA, USA) with 10% FBS (Gibco), 5 mM L-glutamine, 100 U/ml penicillin and 100 μg/ml streptomycin. The medium was placed at 37°C saturated humidity and changed every 2 days. The cells were processed with LPS (SMB00610-1 MG, Sigma-Aldrich, USA) for 24 h at the concentrations (0, 0.1, 1 and 10 μg/ml).

For transfection, cells were cultured in the aforementioned medium at 37°C overnight to reach 70–80% confluence, and then transfected separately with OIP5-AS1 overexpression plasmid (1.5 µg/well) or miR-92a-3p mimic (50 nM). The EcoRI-EcoRI fragment containing full-length cDNA of lncRNA-OIP5-AS1 was inserted into a pIRES2-EGFP vector (Clontech Laboratories, Inc.) to establish lncRNA-OIP5-AS1 overexpression vectors [23]. After 48 h transfection, cells were collected for subsequent experiments. The sequence of miR-92a-3p and the corresponding negative control (NC) were as follows: miR-92a-3p mimic, 5’-UAUUGCACUUGUCCCGGCCUGGGCCGGGACAAGUGCAAUAUU-3’; and miR-NC, 5’-UUCUCCGAACGUGUCACGUTT-3’.

### Reverse transcription-quantitative (RT-qPCR)

Total RNA was subjected to isolation from hPDLSCs with the RNA Isolation kit (Tiangen Biotech Co., Ltd.). Determination of RNA quantification was undertaken with a NanoDrop 2000 spectrophotometer (NanoDrop Technologies). Reverse transcription of RNA to cDNA was done as instructed in the reverse transcription kit (Yeasen Biotech). A standard SYBR Green PCR kit (Takara Bio, Inc.) was used to amplify target fragments. The cDNA fragments of the GAPDH and U6 genes were employed for internal controls. The sequences of designed primer were clearly listed in Table 1. Calculation of individual relative RNA levels was done utilizing the 2^−ΔΔCq^ method [24].

**Table 1.** The primer sequences for RT-qPCR used in the study

Name	Sequences
OIP5-AS1	Forward 5’-TGCGAAGATGGCGGAGTAAG-3’ Reverse 5’-TAGTTCCTCTCCTCTGGCCG-3’
OCN	Forward 5’-CCCAGGCGCTACCTGTATCAA-3’ Reverse 5’-GGTCAGCCAACTCGTCACAGTC-3’
OPN	Forward 5’-AGACCTGACATCCAGTACCCTG-3’ Reverse 5’-GTGGGTTTCAGCACTCTGGT-3’
RUNX2	Forward 5’-TCCACACCATTAGGGACCATC-3’ Reverse 5’-TGCTAATGCTTCGTGTTTCCA-3’
BMP2	Forward 5’-AACACTGTGCGCAGCTTCC-3’ Reverse 5’-CTCCGGGTTGTTTTCCCAC-3’
GAPDH	Forward 5’-ACAACTTTGGTATCGTGGAAGG-3’ Reverse 5’-GCCATCAGCCACAGTTTC-3’
miR-92a-3p	Forward 5’-CGCGTATTGCACTTGTCCC-3’ Reverse 5’-AGTGCAGGGTCCGAGGTATT-3’
U6	Forward 5’-ATTGGAACGATACAGAGAAGATT-3’ Reverse 5’-GGAACGCTTCACGAATTTG-3’

### MTT assay

MTT assay was conducted to determine cell proliferation [25]. The hPDLSCs (2x10^3^ cells/well) processed by LPS were plated into 96-well plates followed by 6 h incubation at 37°C. A total of 20 µl MTT solution at a concentration of 5 mg/ml (cat. no. M-2128; Sigma-Aldrich) was employed to incubate the cells for 4 h at 37°C. Afterward, cells were subjected 15 min incubation at room temperature applying 10 µl DMSO. Finally, the OD value (490 nm) was verified with the aid of a spectrophotometer (Sigma-Aldrich).

### Alkaline phosphatase (ALP) staining

The transfected hPDLSCs were maintained in six-well plates (1x10^4^ cells/well) and treated with 10 μg/ml LPS for 24 h. The cells then were subjected to osteogenic stimulation for 10 days and fixed with 4% paraformaldehyde for 10 min and stained using a Cell Alkaline Phosphatase Activity Stain kit (Genmed Scientifics, Inc.) strictly based on the standard procedures supplied by manufacturer. ALP staining was viewed with the help of an inverted microscope (magnification, x100; Olympus Corporation) [26].

### Biochemical measurements

The transfected hPDLSCs were seeded into six-well plates (1x104 cells/well), followed by treatment with 10 μg/ml LPS for 24 h. The levels of inflammatory cytokines TNF-α (cat. no. ab181421; Abcam), IL-6 (cat. no. ab178013; Abcam) and IL-1β (cat. no. ab214025; Abcam) were detected in cell culture supernatants using the corresponding ELISA kits in keeping with the directions recommended by the supplier [27].

The expression levels of malondialdehyde (MDA) and lactate dehydrogenase (LDH) in the cell lysate were determined separately using an MDA assay kit (cat. no. A003-4-1) and an LDH assay kit (cat. no. A020-2-2). Both reagents were supplied by Nanjing Jiancheng Bioengineering Institute. Following the measurement of either MDA or LDH, the OD was verified at 530 nm by the use of a microplate reader (Sigma-Aldrich).

### Dual-luciferase reporter assay

The OIP5-AS1 wild-type (WT) and mutant (mut) untranslated region (3’-UTR) containing the miR-92a-3p binding site were constructed and subcloned into the pGL3 basic plasmid (Addgene, Inc.). Then, 293 T cells were grown in 24-well plates and incubated at 37°C. Subsequently, the miR-92a-3p mimic and miR-NC were co-transfected into 293 T cells with pGL3-WT or mut-OIP5-AS1 for 48 h. The cells were lysed, and the firefly luciferase activity was measured and normalized to Renilla luciferase activity with the adoption of a Dual-Luciferase Reporter assay system (Promega Corporation) as per the operating protocols.

### RNA immunoprecipitation (RIP) assay

RIP assay was performed to explore the interaction between OIP5-AS1 and miR-92a-3p. Cells were lysed in complete RIP lysis buffer and incubated with magnetic bead–antibody complex overnight at 4°C. The complex was separately detached with proteinase K to extract RNA for subsequent RT-qPCR detection. The RNA concentration was measured by a spectrophotometer (NanoDrop, Thermo Scientific, Waltham, MA, USA), and the RNA quality was assessed using a bioanalyzer (Agilent, Santa Clara, CA, USA).

### Western blotting assay

Following transfection and stimulation with LPS for 24 h, total protein was extracted from hPDLSCs using RIPA lysis buffer containing protease/phosphatase inhibitor cocktail. Total protein was quantified using a BCA protein assay kit (Solarbio Science and Technology Co., Ltd.). An equal amount of protein per lane (25 µg) was separated using an SDS-PAGE gel, transferred to PVDF membranes and subjected to incubation along with primary antibodies against anti-osteocalcin (OCN) (1:1,000; cat. no. ab93876; Abcam), anti-osteopontin (OPN) (1:1,000; cat. no. ab8448; Abcam), anti-runt-related transcription factor 2 (RUNX2) (1:1,000; cat. no. ab76956; Abcam) and anti-bone morphogenetic protein (BMP2) (1:1,000; cat. no. ab14933; Abcam). Subsequently, the incubation of membranes and HRP-conjugated goat anti-rabbit IgG (1:2,000; cat. no. ab6721; Abcam) was carried out. The visualization of protein bands was undertaken with the application of a Tanon-5200 Chemiluminescence Imager (Tanon Science and Technology, Co., Ltd.). The band density was subjected to analysis employing ImageJ software v1.8.0 developed by the National Institutes of Health [28].

### Statistical analysis

All data were presented in the way of mean ± SD of a minimum of three replicates and analyzed adopting SPSS version 23.0 (IBM Corp.). Analysis of variance among multiple groups was conducted by means of one-way ANOVA followed by Bonferroni post hoc test. A probability level of 0.05 was selected showing that the results were significant.

## Results

In this study, we investigated the biological roles of OIP5-AS1 and the potential mechanism in LPS-stimulated hPDLSCs. The results revealed that the overexpression of OIP5-AS1 promoted the proliferation and osteogenic differentiation, but inhibited the inflammatory response under LPS stimulation. Moreover, miR-92a-3p was proved to be sponged with OIP5-AS1. miR-92a-3p overexpression reversed the effects of OIP5-AS1 on LPS-induced hPDLSCs.

### OIP5-AS1 is expressed at low levels in LPS-stimulated hPDLSCs

Aiming to understand the function of OIP5-AS1 in periodontitis, a periodontitis model was established in vitro by inducing hPDLSCs with different concentrations of LPS. In Figure 1 the expression of OIP5-AS1 decreased with increasing LPS concentration, suggesting that OIP5-AS1 may be associated with inflammation in periodontitis. Treatment of 10 μg/ml LPS resulted in lower expression of OIP5-AS1 in hPDLSCs, thus we chose 10 μg/ml LPS for the following experiments.

**Figure 1.** OIP5-AS1 was poorly expressed in LPS-stimulated hPDLSCs. OIP5-AS1 expression in hPDLSCs was assayed by use of RT-qPCR. Error bars indicate the mean ± SD of three-independent replicate experiments. **P < 0.01, ***P < 0.001.

### OIP5-AS1 overexpression promotes the proliferation of hPDLSCs following LPS treatment

The role of OIP5-AS1 in periodontitis was investigated following transfection of hPDLSCs with the OIP5-AS1 overexpression plasmid. RT-qPCR demonstrated that the RNA level of OIP5-AS1 was upregulated in the overexpression (Oe)-OIP5-AS1 group compared with the control group (Figure 2(a)). This result indicated the successful establishment of OIP5-AS1 overexpression. The findings showed that LPS treatment markedly decreased cell proliferation, while OIP5-AS1 overexpression successfully prevented the LPS-induced loss of cell proliferation (Figure 2(b)). The cell shape photographs were shown in Supplemental Figure S1.

**Figure 2.** OIP5-AS1 overexpression promoted the proliferation of hPDLSCs under LPS stimulation. (a) OIP5-AS1 expression in hPDLSCs was examined with the use of RT-qPCR. Error bars indicate the mean ± SD of three-independent replicate experiments. ***P < 0.001. (b) The proliferation of hPDLSCs was assessed with the application of MTT assay. Error bars indicate the mean ± SD of three-independent replicate experiments. ***P < 0.001 vs. Control. ^#^P < 0.05, ^##^P < 0.01, ^###^P < 0.001 vs. LPS.

### OIP5-AS1 overexpression promotes the osteogenic differentiation of hPDLSCs following LPS treatment

To look further into the action of OIP5-AS1 in periodontitis, an ALP staining assay was used to determine the osteogenic differentiation of hPDLSCs following OIP5-AS1 overexpression. Figure 3(a) set up that ALP activity was decreased in the LPS group, but was markedly increased in the LPS + Oe-OIP5-AS1 group. Low expressions of RUNX2 and osteogenic proteins OCN, OPN and BMP2 were found in the LPS group (vs Control). On the other hand, high expressions of RUNX2 and osteogenic proteins were found in the LPS + Oe-OIP5-AS1 group in comparison with the LPS group (Figure 3(b,c)). These results in this section suggested that OIP5-AS1 overexpression promoted the osteogenic differentiation of hPDLSCs following LPS treatment.

**Figure 3.** OIP5-AS1 overexpression promoted the osteogenic differentiation of hPDLSCs under LPS stimulation. (a) The detection of Alkaline phosphatase (ALP) activity was carried out employing ALP staining. Scale bar: 50 μm. (b) The mRNA levels of OCN, OPN, RUNX2 and BMP2 were quantified with RT-qPCR. (c) The protein expressions of OCN, OPN, RUNX2 and BMP2 were examined with the utilization of western blotting. Error bars indicate the mean ± SD of three-independent replicate experiments. **P < 0.01, ***P < 0.001.

### OIP5-AS1 overexpression inhibits the LPS-induced inflammatory response in hPDLSCs

The effect of OIP5-AS1 overexpression on LPS-induced inflammation in hPDLSCs was analyzed using commercial assay kits. Figure 4(a,b) exhibited that LPS elevated the levels of TNF-α, IL-6 and IL-1β, and the expression levels of MDA and LDH in hPDLSCs. However, OIP5-AS1 overexpression markedly suppressed the levels of inflammatory cytokines, MDA and LDH. These evidence presented in this section revealed that OIP5-AS1 overexpression suppressed the LPS-induced inflammation in hPDLSCs.

**Figure 4.** OIP5-AS1 overexpression inhibited the LPS-induced inflammation in hPDLSCs. (a) The levels of TNF-α, IL-6 and IL-1β were assayed with the utilization of ELISA kits. (b) The levels of MDA and LDH were measured by commercial assay kits. Error bars indicate the mean ± SD of three-independent replicate experiments. ***P < 0.001.

### OIP5-AS1 directly targets miR-92a-3p

To investigate the specific molecular mechanisms underlying OIP5-AS1 in LPS-induced inflammation in hPDLSCs, the miRNA-lncRNA interactions were predicted using the Starbase database. The results suggested that OIP5-AS1 directly targeted miR-92a-3p (Figure 5(a)). Furthermore, miR-92a-3p expression was increased with the improvement of LPS concentration (Figure 5(b)). The results of the dual-luciferase reporter and RIP assays demonstrated that OIP5-AS1 directly targeted miR-92a-3p (Figure 5(c,d)). Moreover, RT-qPCR demonstrated that OIP5-AS1 overexpression significantly suppressed miR-92a-3p expression levels (Figure 5(e)). These results suggested that OIP5-AS1 overexpression directly targeted and downregulated miR-92a-3p expression.

**Figure 5.** OIP5-AS1 overexpression directly targeted miR-92a-3p and downregulated its expression. (a)The binding site of OIP5-AS1 and miR-92a-3p. (b) The miR-92a-3p mRNA level was quantified with RT-qPCR. (c) The association between OIP5-AS1 and miR-92a-3p was determined making use of luciferase activity assays. (d) OIP5-AS1 binding to miR-92a-3p detected by RIP assay. (e) The miR-92a-3p mRNA level was quantified with RT-qPCR. Error bars indicate the mean ± SD of three-independent replicate experiments. ***P < 0.001.

### miR-92a-3p overexpression reverses the effect of OIP5-AS1 on the proliferation and osteogenic differentiation of hPDLSCs

To identify the mechanisms underlying OIP5-AS1 in periodontitis, the osteogenic differentiation of hPDLSCs was detected following miR-92a-3p overexpression by transfection with the miR-92a-3p mimic (Figure 6(a)). Cell proliferation was markedly decreased in the LPS + Oe-OIP5-AS1 + miR-92a-3p mimic group compared with the LPS + Oe-OIP5-AS1 group at the indicated time (Figure 6(b)). The cell shape photographs were shown in Supplemental Figure S2. Moreover, miR-92a-3p overexpression partly abolished the facilitative effect of OIP5-AS1 overexpression on the osteogenic differentiation of LPS-stimulated hPDLSCs (Figure 6(c)). The protein and mRNA levels of RUNX2 and osteogenic proteins, OCN, OPN and BMP2 were downregulated by miR-92a-3p overexpression in LPS-stimulated hPDLSCs transfected with Oe-OIP5 (Figure 6(d,e)). These results indicated that miR-92a-3p overexpression reversed the effect of OIP5-AS1 overexpression on the proliferation and osteogenic differentiation of hPDLSCs.

**Figure 6.** miR-92a-3p upregulation reversed the effect of OIP5-AS1 on the proliferation and osteogenic differentiation of hPDLSCs. (a) The miR-92a-3p mRNA level was quantified with RT-qPCR. (b) The assessment of the proliferation in hPDLSCs was conducted employing MTT assay. (c) ALP activity was subjected to analysis with the aid of ALP staining. Scale bar: 50 μm. (d) The mRNA levels of OCN, OPN, RUNX2 and BMP2 were quantified with RT-qPCR. (e) The expressions of osteogenic differentiation markers OCN, OPN, RUNX2 and BMP2 were examined with the adoption of western blotting. Error bars indicate the mean ± SD of three-independent replicate experiments. ***P < 0.001.

### miR-92a-3p overexpression reverses the effect of OIP5-AS1 on LPS-induced inflammation in hPDLSCs

The potential effects of the interaction between miR-92a-3p and OIP5-AS1 on LPS-induced inflammation in hPDLSCs were investigated. It was easily observed in Figure 7(a) that the levels of TNF-α, IL-6 and IL-1β, and the content of MDA and LDH were increased by miR-92a-3p overexpression compared with the LPS + Oe-OIP5-AS1 group (Figure 7(b)). These results indicated that miR-92a-3p overexpression reversed the effect of OIP5-AS1 overexpression on LPS-induced inflammation in hPDLSCs.

**Figure 7.** miR-92a-3p upregulation reversed the effect of OIP5-AS1 on LPS-induced inflammation in hPDLSCs. (a) The levels of TNF-α, IL-6 and IL-1β were assayed with the help of ELISA kits. (b) The levels of MDA and LDH were measured by commercial assay kits. Error bars indicate the mean ± SD of three-independent replicate experiments. ***P < 0.001.

## Discussion

Periodontitis is a chronic non-communicable disease that seriously affects human oral health. Despite extensive studies on the development of periodontitis, very little is currently known about the pathogenesis of periodontitis. PDLSCs are a major cell type of the periodontal tissue with a multi-directional differentiation potential. Moreover, PDLSCs maintain periodontal homeostasis by reshaping and regenerating periodontal tissues [29]. LPS is a potent stimulator of inflammation, can produce proinflammatory cytokines such as TNFα, IL-6, and IL-1β, resulting in disturbance of periodontal ligament cell differentiation, and further leads to deep periodontal tissue destruction and periodontitis [30]. Besides, previous studies also reported that other inflammatory stimuli including may regulate OIP5-AS1 or miR-92a-3p expression [31–34].

The results of previous studies have suggested that lncRNAs are implicated in the development of various inflammatory diseases [14,35,36]. Furthermore, a previous study reported that the expression levels of OIP5-AS1 were low in periodontitis samples compared with healthy subjects [18]. However, the mechanisms that underpin OIP5-AS1 in periodontitis are not fully understood. Zhi et al [37] revealed that OIP5-AS1 was downregulated in osteoarthritis tissues and cellular models, and overexpression of OIP5-AS1 facilitated the malignant behaviors of chondrocyte cells. The results of the present study demonstrated a decreased level of OIP5-AS1 induced by LPS in a concentration-dependent manner, suggesting a latent association between OIP5-AS1 and inflammation in periodontitis. To determine whether OIP5-AS1 expression levels affected the development of periodontitis in a microinflammatory environment, the role of OIP5-AS1 in the proliferation and osteogenic differentiation of LPS-simulated hPDLSCs was examined. This study revealed that OIP5-AS1 overexpression facilitated the proliferation and osteogenic differentiation of hPDLSCs following LPS treatment. Moreover, OIP5-AS1 overexpression suppressed the inflammation in hPDLSCs induced by LPS. Thus, OIP5-AS1 may act as a negative regulator of periodontal inflammation and protect against inflammation in hPDLSCs.

To investigate the specific molecular mechanisms underlying OIP5-AS1 in LPS-induced inflammation in hPDLSCs, the miRNAs that OIP5-AS1 targets were predicted using the Starbase database. The evidence illustrated that miR-92a-3p is a putative target for OIP5-AS1. Furthermore, the findings indicated that OIP5-AS1 directly targeted miR-92a-3p, and OIP5-AS1 overexpression downregulated miR-92a-3p expression. Thus, miR-92a-3p may act as a mediator for OIP-AS1 in hPDLSC proliferation, differentiation and inflammation. Then, we chose miR-92a-3p, the one miRNA that was reported to be associated with periodontitis, to identify the interaction between the miRNA and OIP5-AS1. It is well documented that miR-92a-3p participates in inflammatory responses related to multiple types of diseases [33]. Wang et al [38] showed that miR-92a contributed to the cardiovascular disease development in diabetes mellitus through NF-kappaB and downstream inflammatory pathways. Wiese et al [39]reported that renal injury upregulated endothelial miR-92a-3p expression levels in mice, and inhibition of endothelial miR-92a-3p and miR-489-3p attenuated renal injury-associated atherosclerosis. Kong et al [40] suggested that the increase in miR-92a-3p expression levels in knee osteoarthritis may be involved in inflammation-related processes. In the present study, miR-92a-3p expression were elevated by LPS, which was in line with the results of the aforementioned studies. Interestingly, miR-92a-3p overexpression attenuated the effects of Oe-OIP5-AS1 on the proliferation and osteogenic differentiation of hPDLSCs. Furthermore, miR-92a-3p overexpression reversed the inhibitory effect of OIP5-AS1 overexpression on LPS-induced inflammation in hPDLSCs. Collectively, the results of the present study revealed that OIP5-AS1 inhibited the LPS-induced inflammatory response and promoted the osteogenic differentiation of hPDLSCs by sponging miR-92a-3p. However, due to the aim of this study to explore the role of lncRNA OIP5-AS1 and miR-92a-3p and the molecular mechanism underlying the regulation of lncRNA OIP5-AS1 in periodontitis by targeting miR-92a-3p, we did not investigate the signaling pathways associated with OIP5-AS1/miR-92a-3p in periodontitis. In addition, miR-92a-3p may regulate cell differentiation and inflammation through other lncRNAs in addition to OIP5-AS1, but we here try to study the role of OIP5-AS1/miR-92a-3p in cell differentiation and inflammation of LPS-induced hPDLSCs. We will study the potential pathways of miR-92a-3p and the interactions between miR-92a-3p and other lncRNAs in periodontitis in further study. Besides, we did not study the effect of OIP5-AS1 or miR-92a-3p under non-inflammatory conditions and the effects of downregulation of OIP5-AS1 or miR-92a-3p on osteogenesis or cell proliferation, which will be our future research direction.

## Conclusion

In conclusion, OIP5-AS1 overexpression facilitated the osteogenic differentiation of hPDLSCs and inhibited LPS-induced inflammation. Furthermore, OIP5-AS1 directly targeted and downregulated miR-92a-3p expression, and overexpression of miR-92a-3p expression reversed the effects of OIP5-AS1 on the proliferation and osteogenic differentiation and the LPS-induced inflammation in hPDLSCs.

## Supplementary Material

Supplemental Material
